# PKC*δ* Promotes High Glucose Induced Renal Tubular Oxidative Damage via Regulating Activation and Translocation of p66Shc

This article has been retracted.

**DOI:** 10.1155/2014/746531

**Published:** 2014-10-13

**Authors:** Panai Song, Shikun Yang, Li Xiao, Xiaoxuan Xu, Chengyuan Tang, Yuyan Yang, Mingming Ma, Jiefu Zhu, Fuyou Liu, Lin Sun

**Affiliations:** Department of Nephrology, The Second Xiangya Hospital, Central South University, Changsha, Hunan 410000, China

## Abstract

Diabetic kidney disease (DKD) is a leading cause of end-stage renal disease (ESRD). Renal tubular injury by overproduction of ROS in mitochondria plays a critical role in the pathogenesis of DKD. Evidences have shown that p66Shc was involved in renal tubular injury via mitochondrial-dependent ROS production pathway, but little is known about the upstream signaling of p66Shc that leads to tubular oxidative damage under high glucose conditions. In this study, an increased PKC*δ* and p66Shc activation and ROS production in renal tissues of patients with diabetic nephropathy were seen and further analysis revealed a positive correlation between the tubulointerstitial damage and p-PKC*δ*, p-p66Shc, and ROS production. In vitro, we investigated the phosphorylation and activation of p66Shc and PKC*δ* during treatment of HK-2 cells with high glucose (HG). Results showed that the activation of p66Shc and PKC*δ* was increased in a dose- and time-dependent manner, and this effect was suppressed by Rottlerin, a pharmacologic inhibitor of PKC*δ*. Moreover, PKC*δ* siRNA partially blocked HG-induced p66Shc phosphorylation, translocation, and ROS production in HK-2 cells. Taken together, these data suggest that activation of PKC*δ* promotes tubular cell injury through regulating p66Shc phosphorylation and mitochondrial translocation in HG ambient.

## 1. Introduction

Diabetic kidney disease (DKD) is a leading cause of morbidity and mortality, and it invariably results in an end-stage renal disease (ESRD) [1, 2]. More recently, it has been increasingly documented that the renal tubular injury plays an integral role in the pathogenesis of DKD. In addition, tubulointerstitial lesions are found to be the early and independent features of DKD [3, 4]. Tubular cells injury involves complex etiological and pathophysiological processes. Growing evidence has shown that reactive oxygen species- (ROS-) mediated damage plays a key role in this pathogenesis process affecting renal tubular cells [5–7].

Mitochondrial electron transport chain is the main source of intercellular ROS production [8]. It has been well established that mitochondrial dysfunction participates in the pathological change in tubular injury in DKD [9]. p66Shc, an adaptor protein, is involved in regulation of cellular responses to oxidative stress [10] and is recognized as a new mediator of mitochondrial dysfunction in renal tubular cells under oxidative stress [11–13]. Recent studies demonstrated that p66Shc is phosphorylated at Ser36 residue by apoptosis stimuli and then translocates to the mitochondrial intermembrane space to oxidize cytochrome c, which causes excessive generation of ROS in mitochondria and leads to mitochondrial depolarization [8]. Previous studies in our laboratory have shown that overexpression of a dominant-negative mutant p66Shc (p66Shc S36A) or p66Shc siRNA attenuated or reversed ROS production of mitochondria and cells apoptosis in HK-2 cells, after exposure to angiotensin II or high glucose (HG) ambience [12]. In addition, Pinton et al. [14] found that protein kinase C (PKC)*β*, an isoform of protein kinase C, could induce phosphorylation of p66Shc and triggers mitochondrial accumulation of the protein following activation by oxidative stress. However, whether other isoforms of PKC are also activated and induce mitochondrial translocation of p66Shc in HK-2 cells induced by HG remains unclear.

PKC*δ* is another pivotal member of protein kinase C, a super-family of serine/threonine kinases, which are involved in many signaling pathways to regulate growth, metabolism, differentiation, and apoptosis. PKC*δ* is widely expressed in mammalian tissues, including epithelium, placenta, uterus, brain, and kidney [15], and regulates apoptosis in response to a variety of stimuli including hydrogen peroxide (H_2_O_2_), HG, ultraviolet (UV) radiation, anticancer agents, and ROS [10, 16]. What is more, tyrosine phosphorylation and intracellular translocation of PKC*δ* are responsible for its proapoptotic role in cell oxidative damage state [17, 18]. It is very interesting that the phosphorylated PKC*δ* can bind to p66Shc in COS-7 cells induced by H_2_O_2_ stimulation, which may play a critical role in the oxidative stress signaling pathway [19]. Hence, we speculate that PKC*δ* may associate with p66Shc and participates in oxidative damage in renal tubular cells in DKD. However, the role of PKC*δ* on p66Shc activation and mitochondrial translocation in HK-2 cell exposed to HG is not fully understood. In this study, we aimed to assess the expression of p-p66Shc and p-PKC*δ* in renal tissues of patients with DKD and analyzed the relationship between their expressions and kidney oxidative injury in vivo. We also assessed the role of PKC*δ* in regulating p66Shc activation and mitochondrial translocation in HK-2 cells induced by HG.

## 2. Materials and Methods

### 2.1. Main Reagents and Materials

Human proximal tubular epithelial cells (HK-2) were purchased from ATCC American. Antibodies were obtained from the following sources: polyclonal anti-PKC*δ* and polyclonal anti-phospho-PKC*δ*-Tyr-311 from Cell Signaling Technology (Boston, MA) and monoclonal anti-p66Shc and monoclonal anti-phospho-p66Shc-S36 from Abcam (USA). All secondary antibodiesfor Western blot analysis were from ZSGB-BIO (Beijing, China), and secondary antibodies for immunofluorescence were from Jackson ImmunoResearch (West Grove, PA). Rottlerin was obtained from Enzo life sciences (USA), mitochondria isolation kit was purchased from Beyotime (Jiangsu, China), 4′,6-diamidino-2-phenylindole 9 (DAPI) was from Sigma-Aldrich (St. Louis, MO), PKC*δ* siRNA (h) was from Santa Cruz (USA), Lipofectamine 2000 and MitoSOX were from Invitrogen (USA), 2,7-dichlorodihydrofluorescein diacetate (DCFH-DA) and dihydroethidium (DHE) were from Sigma-Aldrich (USA), and DAB kit was from CWBIO (Beijing, China). Other reagents, including DMEM medium with low glucose (1000 mg/L), bovine serum albumin (FBS), and trypsin, were obtained from GIBCO (USA).

### 2.2. Morphological Evaluation of Kidney

Human renal biopsy tissues from 32 cases (16 with DN and 16 with minimal change nephropathy) were studied by special stain (PAS and PASM) to assess glomerular, tubulointerstitial pathological change. A semiquantitative scoring system was used to evaluate the severity of tubulointerstitial injury [20, 21]. The human experimental procedures as described above were approved in advance by the Institutional Human Experimentation Ethics Committee, The Second Xiangya Hospital, Central South University.

### 2.3. Immunohistochemistry (IHC)

Renal tissue sections for immunostaining were deparaffinized, rehydrated, and blocked with 3% H_2_O_2_ solution, followed by antigen retrieval in a microwave oven. The sections were then incubated with antibodies directed against phospho-PKC*δ*-Tyr-311 (1 : 50) and phospho-p66Shc-Ser36 (1 : 100), respectively, and visualized by using a DAB detection kit according to the manufacturer's instructions. Slides were mounted with coverslip and examined with a Zeiss fluorescence microscope. Intracellular generation of O_2_^−^ was assessed by DHE staining.

### 2.4. HK-2 Cell Culture and Treatment

HK-2 cells were cultured in DMEM medium supplemented with 10% FBS, penicillin 1 × 10^5^ U/L, and streptomycin 100 mg/L and incubated at 37°C in a 5% CO_2_ environment until the cells were 80% confluent. Cells were then incubated in DMEM medium without FBS for 24 hrs. HK-2 cells were cultured with different concentrations of D-glucose (5 mM–30 mM) for 24 hrs or with 30 mM D-glucose only for indicated time points (0 min–180 min); then, the expression of PKC*δ* and p66Shc and phosphorylation of both PKC*δ* (p-PKC*δ*) and p66Shc (p-p66Shc) were detected by western blotting and immunofluorscence, respectively. In addition, the effect of PKC*δ* on the phosphorylation and mitochondrial translocation of p66Shc in HK-2 cells exposed to HG was also observed by isolation of mitochondria from HK-2 cells for Western blot analysis.

### 2.5. Small Interfering RNA for PKC*δ*

Human small interfering RNA (siRNA) for PKC*δ* and scrambled siRNA were obtained by Santa Cruz (Santa Cruz, USA). The targeted sequences to silence the transcription of human PKC*δ* were 5′-GUC UGG UAA GAC UGG AGU ACC-3′. The PKC*δ* siRNA (final concentration at 20 nM) and scrambled siRNA were transfected into the HK-2 cells according to manufacturer's instructions.

### 2.6. Western Blot Analysis

The total protein of HK-2 cells was extracted with RIPA lysis buffer which contains protease inhibitors. Following the vendor's instructions, mitochondrial and cytosolic proteins were individually isolated from HK-2 cells by using a mitochondrial isolation kit. The protein expressions of total p66Shc and PKC*δ* as well as p-p66Shc and p-PKC*δ* were assessed using anti-p66Shc, anti-PKC*δ*, anti-p-p66Shc (Ser36 site), and anti-p-PKC*δ* (Tyr311 site). The antimitochondrial Cox IV antibody was used as loading controls for mitochondrial fractions. The anti-*β*-actin was used for loading controls of cytoplasm fractions. Western Blot Kit (with HRP conjugated rabbit or mouse secondary antibody) was used for visualizing the bands.

### 2.7. Immunofluorescence Staining

For cell staining, HK-2 cells were seeded on glass slides. Cells were fixed with 4% paraformaldehyde (PFA) for 15 min and then washed in PBS (three times, 5 min each). For staining of p-p66Shc and p-PKC*δ*, cells were treated with 0.1% Triton X-100 for 10 minutes and with blocking buffer containing 10% normal goat serum for half an hour at room temperature, and then the cells were incubated in primary antibody solution overnight (anti-p-p66Shc, 1 : 50, and anti-p-PKC*δ*, 1 : 100). Fluorochrome-conjugated secondary antibodies (diluted 1 : 400 in PBS containing 5% BSA) were used for incubating cells for 1 hour at room temperature. DAPI was used to stain the nuclei.

### 2.8. Detection of Intracellular H_2_O_2_ and Assessment of Mitochondrial Superoxide Anion (O_2_^∙−^)

The dichlorofluorescein diacetate (DCFH-DA), a H_2_O_2_-sensitive fluorescence probe, was applied to assess the intracellular H_2_O_2_, as previously discussed [8, 22]. MitoSOX Red (Invitrogen), a live-cell permeant dye that rapidly and selectively targets mitochondria, was used to observe mitochondrial O_2_^∙−^. The DCFH-DA fluorescence (with excitation at 490 nm and emission at 520 nm) and MitoSOX red fluorescence (with excitation at 510 nm and emission at 585 nm) were detected in a laser scanning confocal microscope equipped with band-pass filter (Zeiss LSM 510; Carl Zeiss, Thornwood, NY). After staining with DCFH-DA and MitoSOX Red, intracellular H_2_O_2_ and mitochondrial O_2_^∙−^ were also detected by FACS analysis [22].

### 2.9. Data Analysis

Statistical analysis was carried out using the SPSS16.0 software. The experimental results were expressed as mean values ± standard error of the mean (SEM). One-way ANOVA was used to analyze the differences among groups, and two-tailed *P* values are reported. A value of *P* < 0.05 was considered statistically significant.

## 3. Results

### 3.1. Increased p-PKC*δ* and p-p66Shc Expression and ROS Production in Renal Tissues of Patients with Diabetic Nephropathy (DN)

PAMS and PAS staining revealed obvious changes in the morphology of both glomerular and tubulointerstitial compartments; they included focal tubular atrophy and interstitial fibrosis in DN patients (Figure 1(a) ((A)–(D)) and Figure 1(e)). IHC staining revealed notable increased p-PKC*δ* and p-p66Shc expression in the renal tubules of patients with DN (Figure 1(a) (E)–(H)). In addition, the staining intensity was also increased by >60% in DN patients, as assessed by semiquantitative analyses (Figures 1(b) and 1(c)). ROS production was detected by using ROS-sensitive vital dye dihydroethidium, which revealed increased ROS generation in kidney tissues of DN patients (Figure 1(a) ((I)-(J)) and Figure 1(d)). Further analysis revealed a positive correlation between the tubulointerstitial damage and p-PKC*δ* and p-p66Shc expression and ROS production (Figure 1(f)).

### 3.2. HG Induced Phosphorylation of PKC*δ* and p66Shc in HK-2 Cells

HK-2 cells were exposed to different concentrations of D-glucose (5 mM–45 mM) for 120 min; then, protein expression and phosphorylation of PKC*δ* and p66Shc were determined by Western blotting analyses. As shown in Figure 2(a), there was no obvious change in protein expression of total PKC*δ* and p66Shc (middle panels), while the phosphorylated PKC*δ* (Tyr311) and p66Shc (Ser36) were significantly increased in a dose-dependent manner in HK-2 cells treated with HG (upper panels). In addition, HK-2 cells were treated with D-glucose (30 mmol/L) for various times (0 min–180 min). Results indicated that HG induced the phosphorylation of p66Shc (Ser36) and PKC*δ* (Tyr311) in a time-dependent manner within 15 min and expression was sustained for 180 min (Figure 3(a), upper panels). However, no change was observed in total PKC*δ* and p66Shc expression (Figure 3(a), middle panels).

### 3.3. Inhibition of HG-Induced p66Shc Phosphorylation in HK-2 Cells by Rottlerin

To investigate whether PKC*δ* is involved in the activation of p66Shc in HK-2 cells with HG, we initially investigated the toxic effects of Rottlerin, a pharmacologic inhibitor of PKC*δ*, since it has been reported that Rottlerin is toxic to the rat kidney proximal tubular cells when exposed to more than 5.0 *μ*M concentration [23]. We examined the effects of Rottlerin with lower concentrations (0.5 to 4.0 *μ*M) on HK-2 cells prior to 30 mM D-glucose treatment and found that HG induced PKC*δ* activation and it was notably suppressed by Rottlerin in a dose-dependent manner (data not shown). In order to reduce the potential toxicity of Rottlerin to HK-2 cells, we chose 1 *μ*M Rottlerin for this study. We found that 1 *μ*M Rottlerin could significantly inhibit p66Shc phosphorylation in HK-2 cells treated with HG (Figure 4(a), upper panel, lane 3 versus lane 2). No change was seen in the total p66Shc expression (middle panel). Similar results were also observed by cells immunofluorescence staining. As shown in Figure 4(c), HG also increased the phosphorylation of PKC*δ* and p66Shc, while this effect was abolished with the treatment of Rottlerin. These data suggested that PKC*δ* may be involved in HG-induced p66Shc phosphorylation.

### 3.4. Inhibition of HG-Induced p66Shc Phosphorylation in HK-2 Cells by PKC*δ* siRNA

To further ascertain that PKC*δ* is involved in p66Shc phosphorylation in response to HG stimulation, we used RNAi method to knock down endogenous PKC*δ* in HK-2 cells. With PKC*δ* siRNA treatment a marked decrease of p66Shc phosphorylation was seen in the HK-2 cells subjected to HG treatment (Figure 5, lane 4 versus lane 2). No change was found in the levels of p66Shc phosphorylation in HK-2 cells treated with PKC*δ* siRNA compared to that of control siRNA treatment (lane 3 versus lane 1). These results confirmed that PKC*δ* participated in the phosphorylation of p66Shc in HK-2 cells treated with HG.

### 3.5. PKC*δ* Modulates the Mitochondrial Translocation of p66Shc in HK-2 Cells in Response to HG Stimulation

To investigate the mechanisms by which mitochondrial translocation of p66Shc occurs, cells transfected with PKC*δ* siRNA or scrambled siRNA were exposed to 30 mM D-glucose for different time intervals (0 min–180 min). The cytosolic and mitochondrial fractions were then isolated from HK-2 cells for Western blot analysis. As shown in Figure 6(a), compared with control (5 mM D-glucose), markedly increased phosphorylation of p-p66Shc in a time-dependent manner was observed in the cytosolic fractions of HK-2 cells treated by HG (Figure 6(a) upper panels, lanes 2–4 versus lane 1, and Figure 6(b)), while this effect was suppressed by treatment with PKC*δ* siRNA (Figure 6(a) upper panels, lanes 5–7 versus lanes 2–4, and Figure 6(b)). In contrast, the expression of p66Shc was also increased in time-dependent manner in mitochondrial fractions isolated from HK-2 cells treated by HG (Figure 6(a) middle panels, lanes 2–4 versus lane 1, and Figure 6(c)), while this effect was abolished with the treatment of PKC*δ* siRNA (Figure 6(a) middle panels, lanes 5–7 versus lanes 2–4, and Figure 6(c)). Together, the results suggest that the phosphorylation of p66Shc and its mitochondrial translocation in response to HG stimulation is dependent on activity of PKC*δ*.

### 3.6. PKC*δ* siRNA Attenuates the Generation of Intracellular ROS and Mitochondrial Superoxide in HK-2 Cells Subjected to HG

By confocal microscopy, cells stained with DCFH-DA revealed an increase in intracellular ROS production in HK-2 cells treated with HG, while it was reduced with the treatment of PKC*δ* siRNA (Figure 7(a), upper panel). In addition, to measure mitochondrial superoxide (O_2_^∙−^), the MitoSOX Red probe was used. Results showed that HG also increased the mitochondrial O_2_^∙−^ generation, which was also markedly reduced with the treatment of PKC*δ* siRNA (Figure 7(a), lower panel). Similar results were observed by FACS analyses (Figures 7(b) and 7(c)).

## 4. Discussion

The number of pathways and molecules participating in the progression of DKD has been reported, and it is believed that renal proximal tubular cell oxidative damage and apoptosis with the overproduction of ROS are associated with the early stages of DKD [5], and this plays a key role in the progression of DKD [24]. p66Shc is a vital adaptor protein that regulates oxidative stress and life span in mammals cells, and genetic deletion of p66Shc can attenuate hyperglycemia-induced endothelial dysfunction and oxidative damage [25, 26]. Vashistha and Meggs [27] found that p66 null Akita mice have marked attenuation of oxidative stress and glomerular/tubular injury and distinct reduction in urine albumin excretion. This finding indicates that p66Shc-mediated oxidative stress plays a central role in renal oxidative injury of DKD. However, detailed molecular mechanism of p66Shc activation and its mitochondrial translocation in this process need be further addressed.

It is known that p66Shc and its activity are significantly increased in both kidneys of STZ-induced diabetic mice and db/db mice, a type 2 diabetic mice model, which are associated with increased oxidative damage [12]. Moreover, PKC*β* can be activated by hyperglycemia and oxidative stimulus in renal tubular cells and it is accompanied with phosphorylation of p66Shc [8, 14, 28], and inhibition of PKC*β* could partially prevent p66Shc phosphorylation and its mitochondrial translocation in HK-2 cells treated with HG [12]. Furthermore, increased evidence indicates that inhibition of PKC*β*II activation prevents phosphorylation of p66Shc in human aortic endothelial cells exposed to hyperglycemic stress or oxidized low-density lipoprotein and protects mice from gut I/R injury by suppressing the adaptor p66Shc mediated oxidative stress [29–31]. These data indicate that PKC*β*II is an important protein that mediates the phosphorylation of p66Shc in diabetic nephropathy. However, whether other PKC members are also involved in this process is still unknown.

This study demonstrates a significant role for PKC*δ* in tubular cell oxidative damage under hyperglycemic states. First, we discovered that both p66Shc phosphorylation and PKC*δ* phosphorylation were increased in renal proximal tubules of patients with DKD compared with non-DN patients, which apparently induce increased oxidative damage to the tissues (Figure 1). These results support our previous hypothesis: there is a close relationship between the phosphorylation of p66Shc and PKC*δ* activation, and here we further confirmed it by in vitro studies. Results showed that PKC*δ* activation was accompanied with the phosphorylation of p66Shc induced by HG in HK-2 cells (Figures 2 and 3), which is consistent with the results reported by Liu et al. [32] that tyrosine phosphorylation of PKC*δ* can be induced by HG in neural precursor cells. These results indicate that HG can induce activation of PKC*δ*, and p66Shc phosphorylation may be associated with PKC*δ*.

Recent evidence [33] indicates that the formation of PKC*δ*/p66Shc/Cyt.C complex plays a significant role in cellular oxidative damage mediated by PKC*δ*. Knocking out anyone of these genes will disrupt the signaling pathways of oxidative damage. In addition, Morita et al. [19] have discovered that Tyr331 of PKC*δ* was phosphorylated by epidermal growth factor receptor (EGFR) in COS-7 cells with the stimulation of H_2_O_2_, and then it bound with p66Shc and EGFR to form a complex, which played an important role in oxidative stress. Therefore, we speculated that PKC*δ* may play a potential role in tubular cell oxidative damage with p66Shc involvement under HG ambience. In this study, we demonstrated that treatment with Rottlerin, a specific blocker of PKC*δ*, markedly suppressed HG-induced p66Shc phosphorylation (Figure 4). Although Rottlerin has been used in many researches to clarify the role of PKC*δ* in a variety of cellular events, it also inhibits many other protein kinases including p38-regulated/activated kinase, calmodulin-dependent protein kinase III, and mitogen-activated protein kinase-activated protein kinase 2 [15, 34]. Therefore, to assess the role of PKC*δ* in p66Shc phosphorylation, knockdown of endogenous PKC*δ* with RNAi was used in HK-2 cells. Results indicated that PKC*δ* siRNA partially blocked HG-induced p66Shc phosphorylation (Figure 5) and its mitochondrial translocation (Figure 6). Thus, our data strongly indicated that PKC*δ* could modulate p66Shc phosphorylation and its mitochondrial translocation in HK-2 cells exposed to HG ambience. In addition, a study by Lin et al. [35] revealed that PKC*δ*-knockdown selectively decreased expression of PKC*β*II in human macrophages. This data indicated that there may be potential interactions and regulations between PKC*δ* and PKC*β*II. Here we demonstrated that PKC*δ* could induce the phosphorylation of p66Shc in HK-2 cells exposed to HG; whether or not PKC*δ* is involved in this process by regulating PKC*β*II needs to be further studied in future.

Accumulating evidence indicates that PKC*δ* is responsible for elevated intracellular ROS production in HF adipocytes, which is mediated by high glucose and NADPH oxidase [36]. Moreover, PKC*δ* knockout mice reveal reduced ROS formation, and they were resistant to cell death induced by different stimuli [37]. To address whether PKC*δ* participates in the intracellular ROS production by regulating p66Shc phosphorylation and mitochondrial translocation in HK-2 cells following the treatment of HG, DCFH-DA, a dye probe that measures ROS (H_2_O_2_) in the cytosol, and MitoSOX, a mitochondrial superoxide (O_2_^∙−^) indicator, were employed. As elucidated in Figure 7, HG increased intracellular ROS production as well as mitochondrial O_2_^∙−^ generation, and this effect was blocked by overexpression of PKC*δ* siRNA. These observations support that PKC*δ* plays a crucial role in HG-induced mitochondrial ROS production mediated by p66Shc. Furthermore, it has been reported that phosphorylation of p66Shc induced by PKC*β* under oxidative stress states could be isomerized by prolyl isomerase (Pin1), and then it might be dephosphorylated by PP2A. After dephosphorylation, p66Shc translocates into mitochondria, promoting the ROS generation [14]. However, recent studies [38, 39] have suggested that activation of PKC*δ* by oxidative stress results in its mitochondrial translocation, leading to release of cytochrome c and the induction of apoptosis. In addition, Leitges et al. [40] have reported that phosphorylated PKC*δ* binds to the SH2 domain of Shc isoforms in antigen-stimulated mouse bone marrow-derived mast cells. These discoveries indicate that activation of PKC*δ* can lead to phosphorylation of p66Shc and may form a complex with p66Shc, which then translocates to mitochondria. Nevertheless, it remains unknown how PKC*δ* regulates p66Shc during renal tubular cell injury. Our results do not show clear evidence for direct interaction of p66Shc by PKC*δ*. Thus, further studies are required to elucidate the protein interaction of PKC*δ* and p66Shc in the regulation of cell oxidative damage under HG ambience. It would be important to investigate in future to gain in-depth understanding of the regulation of tubular cell injury by PKC*δ* during the mitochondrial pathway.

In recent years, specific inhibitor of PKC*β* has been reported to be used in many experimental models of DKD, which could effectively protect against kidney damage [41]. Moreover, it is currently the focus of clinical trials for several cardiovascular diseases and DKD [42, 43]. Hence, it would be also of great interest to investigate the effects of PKC*δ* inhibitors in DKD. However, studies have indicated that selective inhibitor of PKC*δ*, Rottlerin, was toxic to cells after a certain concentration [23], so large-scale clinical trials will need to validate safety and prospective application of Rottlerin in DKD.

In conclusion, this study has confirmed the increased activation of PKC*δ* as well as p66Shc during HG treatment of renal tubular cells in vitro and hyperglycemia in vivo. Under the experimental conditions, blockade of PKC*δ* pharmacologically or genetically can suppress HG-induced p66Shc phosphorylation and its mitochondrial translocation and protect the cells against oxidative damage. These data suggest that a novel PKC*δ*/p66Shc pathway may be involved in the pathogenesis of oxidative damage in diabetic kidney (Figure 8). Our results may also provide a new treatment strategy by targeting PKC*δ* for renoprotection in diabetic nephropathy or other oxidative stress diseases.

## Figures and Tables

**Figure 1:** Increased p-PKC*δ* and p-p66Shc expression and ROS production in renal tissues of patients with diabetic nephropathy (DN). Renal biopsy samples were collected from 16 of DN patients and 16 of non-DN patients. Tubular atrophy and interstitial fibrosis were seen in renal biopsies in patients with DN as detected by PASM and PAS staining (panels (B) and (D) versus panels (A) and (C)). Immunohistochemical studies revealed increased expression of p-PKC*δ* and p-p66Shc in DN patients (panels (F) and (H) versus panels (E) and (G)) (magnification ×200). Status of oxidant stress in kidneys of DN and non-DN patients indicated in panels (I) and (J). ((b) and (c)) Averaged relative intensity following staining of anti-p-PKC*δ* and anti-p-p66Shc antibody of renal biopsies of DN patients versus non-DN patients. (d) Relative fluorescence intensity of dihydroethidium (DHE) in kidneys of DN and non-DN patients. (e) Tubular interstitial damage score in DN patients versus non-DN patients. (f) Table shows correlation between p-PKC and p-p66Shc expression, DHE level, and tubular interstitial damage. Values are means ± SEM, ^*^ *P* < 0.01.

**Figure 2:** HG induced phosphorylation of PKC*δ* and p66Shc in HK-2 cells in a dose-dependent manner. Protein expression of PKC*δ* and p66Shc and their phosphorylation in HK-2 cells following exposure to HG (5–45 mM) for 120 min were determined by Western blot analysis. 45 mM of D-mannitol as an osmotic control. Phosphorylation of both PKC*δ* and p66Shc increased in a dose-dependent manner in HK-2 cells treated with high glucose. No change was observed in the expression of total protein of PKC*δ* and p66Shc; *β*-actin served as a loading control (a). ((b) and (c)) The bar graphs represent the expression of p-PKC*δ* and p-p66Shc relative to PKC*δ* and p66Shc, respectively. Values are means ± SEM; *N* = 5. ^*^ *P* < 0.05, ^#^ *P* < 0.01 versus control.

**Figure 3:** HG induced phosphorylation of PKC*δ* and p66Shc in HK-2 cells in a time-dependent manner. Expression of PKC*δ* and p66Shc and their phosphorylation in HK-2 cells following exposure to 30 mM HG for indicated time points (0–180 min) were determined by Western blot analysis. Expression of both p-PKC*δ* and p-p66Shc increased in a time-dependent manner in HK-2 cells treated with high glucose, while there was no change in total protein expression of PKC*δ* and p66Shc; *β*-actin served as a loading control (a). ((b) and (c)) The bar graphs represent the expression of p-PKC*δ* and p-p66Shc relative to PKC*δ* and p66Shc, respectively. Values are means ± SEM; *N* = 7. ^*^ *P* < 0.05, ^#^ *P* < 0.01 versus control.

**Figure 4:** Rottlerin inhibits HG-induced p66Shc phosphorylation in HK-2 cells. Cells were treated with Rottlerin for 30 min prior to HG (30 mM) treatment. Total proteins were collected for Western blot analysis of p-p66Shc, total p66Shc, and *β*-actin ((a) and (b)). (c) By immunocytofluorescence microscopy, the increased phosphorylation of PKC*δ* and p66Shc was seen in HK-2 cells after treatment with 30 mM HG, while this effect was significantly attenuated in Rottlerin group. Values are means ± SEM, *N* = 3. ^*^ *P* < 0.01 versus LG group, ^#^ *P* < 0.01 versus HG-only group.

**Figure 5:** PKC*δ* siRNA inhibits HG-induced p66Shc phosphorylation in HK-2 cells. HK-2 cells were transfected with either PKC*δ* siRNA or scrambled siRNA and then stimulated with 30 mM HG for 24 hrs. PKC*δ*, p66Shc, and p-p66Shc were detected by Western blot analysis. An increased expression of p-p66Shc was observed in HK-2 cells induced by HG, but it failed in the group treated with PKC*δ* siRNA. Values are means ± SEM, *N* = 4. ^*^ *P* < 0.01 versus LG group, ^#^ *P* < 0.01 versus scrambled siRNA.

**Figure 6:** PKC*δ* siRNA inhibits p66Shc translocation during HG treatment of HK-2 cells. HK-2 cells were transfected with PKC*δ* siRNA or scrambled siRNA and treated with HG for different time periods. Lysates of cytosolic and mitochondrial fractions were analyzed for p66Shc and p-p66Shc expression by Western blotting, and *β*-actin was used as a cytosolic loading control and Cox IV antibody was used as a mitochondrial loading control. Values are means ± SEM, *N* = 4. ^*^ *P* < 0.01 versus HG group.

**Figure 7:** PKC*δ* siRNA attenuates the generation of intracellular ROS and mitochondrial superoxide in HK-2 cells exposure to HG. (a) HK-2 cells were stained with dichlorofluorescein-diacetate (DCFH-DA) and MitoSOX, respectively, and then examined by confocal microscopy. Results indicate that PKC*δ* siRNA exhibits reduced intracellular ROS production in HK-2 cells after treatment with HG (row 1). Similar results were seen in mitochondrial ROS production as assessed by MitoSOX staining (row 2). ((b) and (c)) The bar graphs represent a summary of flow cytometry analyses of cells stained with DCFH-DA and MitoSOX, respectively. Values are means ± SEM, *N* = 4. ^*^ *P* < 0.01 versus 5 mM D-glucose. ^#^ *P* < 0.01 versus 30 mM D-glucose.

**Figure 8:** Schematic drawing depicting PKC*δ* mediates p66Shc phosphorylation and mitochondrial translocation induced by HG. With treatment of HG, PKC*δ* is activated, promoting p66Shc phosphorylation and its translocation to mitochondria, where p66Shc oxidizes mCyt.C to induce mitochondrial ROS generation, which results in oxidative damage and apoptosis of renal tubular epithelial cells.
